RETRACTED

# Siglec-15 Regulates the Inflammatory Response and Polarization of Tumor-Associated Macrophages in Pancreatic Cancer by Inhibiting the cGAS-STING Signaling Pathway

**DOI:** 10.1155/2022/3341038

**Published:** 2022-09-05

**Authors:** HuaGen Li, RongXuan Zhu, XiaoLong Liu, Kai Zhao, DeFei Hong

**Affiliations:** ^1^School of Medicine, Zhejiang University, 866 Yuhangtang Road, Hangzhou, 310058 Zhejiang, China; ^2^Department of General Surgery, Sir Run Run Shaw Hospital, The Medicine School of Zhejiang University, Hangzhou, China; ^3^Department of Thoracic Surgery, National Cancer Center, National Clinical Research Center for Cancer, Cancer Hospital, Chinese Academy of Medical Sciences and Peking Union Medical College, Beijing, China

## Abstract

Tumor-associated macrophages especially M2 phenotype macrophages play an important role in tumor progression and the formation of immunosuppressive tumor microenvironment. Previous studies indicated that infiltration of a large number of M2-macrophages was positively associated with a low survival rate and poor prognosis of patients with pancreatic ductal cancer. However, the mechanisms responsible for M2-macrophage polarization remain unclear. Recently, Siglec-15 appears as an emerging target for the normalization of the tumor immune microenvironment. Hence, we detected the Sigelc-15 expression on macrophages by using qPCR and Western blot assay and found that the expression of Siglec-15 was upregulated on M2 macrophages induced by IL-4 and conditioned media from pancreatic ductal cancer. In addition, after knocking out Siglec-15, the expression of M2 phenotype macrophage biomarkers such as Arg1 and CD206 was significantly downregulated. Besides, in our study we also found that Siglec-15 could upregulate the glycolysis of macrophage possibly by interacting with Glut1 to regulate the M2-macrophage polarization. The regulation was also partly dependent on STING, and Glut1-related glycose metabolism was involved in regulating cGAS/STING signaling. When utilizing a subcutaneous transplantation mouse model, we observed that knocking out of Siglec-15 or co-injecting tumor cells with macrophage from Siglec-15 KO mice could significantly inhibit the growth of subcutaneous tumors in mice. Taken together, these findings suggest that Siglec-15 is essential for the M2-macrophage polarization to shape an immune suppressive tumor microenvironment in pancreatic cancer and makes it an attractive target for pancreatic cancer immunotherapy.

## 1. Introduction

Pancreatic ductal cancer (PDAC) is one of the most lethal malignancies with a poor prognosis and short overall survival [1]. According to the most recent global tumor statistics, the number of new cases and death cases of PDAC exceeded 400,000 last year. The fact that its occurrence is rising among younger people has a significant negative effect on the quality of life of individuals [2, 3]. Despite the modest improvement in surgical and adjuvant treatment for PDAC, the overall survival of PDAC is only minimally improved with a 5-year survival rate of 8% [4]. Hence, the effective treatments for pancreatic cancer are still urgently needed.

RETRACTED

In recent years, multiple studies have demonstrated that the tumor-immunosuppressive microenvironment had an indispensable impact on the occurrence and development of pancreatic cancer and immunotherapy for PDAC [4–6]. Tumor-associated macrophages (TAMs) which are the most abundant infiltrative immune cells in the tumor microenvironment (TME) play an important role in tumor progression [7]. Generally, macrophages could be polarized into M1 or M2-like phenotype macrophages depending on different environments around it [8]. M1-macrophages are proinflammatory and tumor suppressive, while M2-macrophages are anti-inflammatory and promote tumorigenesis and immunosuppression. However, macrophages located in the tumor microenvironment of PDAC are preferentially polarized into the M2-like phenotype to promote the tumor progression and formation of the immunosuppressive TME [9, 10]. Additionally, it was observed that the infiltration of M2 macrophages was substantially related with tumor metastasis, chemoresistance, and a poor prognosis in a variety of malignancies, including PDAC [11, 12]. Therefore, polarization mechanisms of TAMs have emerged as a focus of intense attention in the field of cancer research and offer the potential for an effective immunotherapy strategy for PDAC.

Sigelc-15 is indicated highly expressed in M2 macrophages and appears as an emerging target for tumor immunotherapy. However, its biological function in TAMs of PDAC remains to be determined. In this study, we found that sialic acid-binding immunoglobulin-like lectin 15 (Siglec-15), which could enhance tumor immune escape in TME without an association with the PD-1/PD-L1 pathway [13–15], played an important role in the polarization of TAMs. Our findings suggest that within the TME of pancreatic cancer, Siglec-15 could promote TAMs to polarize into M2 macrophages and contribute to shaping an immunosuppressive TME to promote tumor progression. In addition, we also found that Siglec-15 regulates polarization of TAMs by upregulating glycolysis of macrophages and the cyclic GMP-AMP synthase (cGAS)-stimulator of interferon genes (STING) signaling pathway as well as Glut1-related glycose metabolism was involved in polarization mechanisms.

RETRACTED

## 2. Methods

### 2.1. Cell Culture and Transfection

Mouse-derived macrophages RAW264.7; pancreatic ductal cancer cell lines BxPC-3, SW1990, and PANC-1; and normal pancreas cell lines H6C7 were purchased from the American Type Culture Collection (ATCC). Bone marrow-derived macrophages (BMDMs) are extracted from mouse bone marrow cells and induced by adding L929-conditioned medium [16]. When the experimental cell density was about 70%, the serum-containing DMEM medium was replaced with a serum-free Opti-MEM medium. Lipofectamine™ 2000 Reagent (Invitrogen) and plasmid were configured using a transfection system based on plasmid DNA quality and Lipofectamine™ 2000 volume 1 : 1. Then, the transfection system was added to the cell culture medium. After six hours, the Opti-MEM medium was replaced with a serum-containing DMEM medium and was cultured at 37°C for one day before further processing.

### 2.2. Polarization of Bone Marrow-Derived Macrophages (BMDMs)

BMDMs with a maturation rate greater than 90% were used in this study. After stimulation with 100 ng/mL LPS and 20 ng/mL IFN-*γ* for 12 h, BMDMs were induced into M1 macrophages [17], while stimulation with 20 ng/mL IL-4 for 24 h induced BMDMs polarized into M2 macrophages. Tumor cell supernatant and DMEM complete medium were made into conditioned medium at 1 : 1 and stimulated BMDMs. The phosphorylation level of biomarkers was detected at different time points.

### 2.3. Real-Time Quantitative PCR (qPCR)

Routinely culture mouse macrophages RAW264.7, adjust the cell density to 2.5 × 10^5^ cells/mL, and maintain them in a 37°C 5% CO_2_ incubator for 24 h. Total RNA was extracted using TRIzol Reagent (Invitrogen, Thermo Fisher Scientific, Inc.) according to the manufacturer's instructions. The mRNA expression was assayed by RT-qPCR. For each sample, 1 *μ*g of RNA was taken for reverse transcription reaction. The reverse transcription product was collected to perform a PCR reaction. RT-qPCR was performed using the Bio-Rad CFX96 real-time system, and the PCR reaction conditions were as follows: 95°C for 30 s, 95°C for 5 s, 60°C for 30 s, 40 cycles [18]. For the analysis of gene expression, gene expression levels were normalized to the expression of GAPDH to calculate the 2^−*ΔΔ*Ct^ value. The primer sequences are shown in Table 1.

### 2.4. Western Blotting

Proteins from cells were extracted with RIPA buffer with 0.1 mmol/L PMSF (Beyotime Biotechnology, Shanghai) and quantified using the BCA kit (Beyotime Biotechnology, Shanghai) [19]. The total protein (20 *μ*g/lane) was separated on 10% SDS-PAGE gel followed by transfer to the PVDF membrane (EMD Millipore, MA, USA). The membrane was blocked in 5% skimmed milk powder at room temperature for 2 h, then incubated with a primary antibody (1 : 1000) overnight at 4°C. After incubating with the primary antibody, the membrane was washed three times with TBST and incubated with a secondary antibody (1 : 2500) for 1 h at room temperature. Protein bands were visualized using the ECL kit (Millipore, USA), and the blots were developed and exposed using a ChemiDoc™ Touch Imaging System. Commercial antibodies used in vitro cultures, and western blots were purchased from Abcam, BD Biosciences, or R&D Systems.

RETRACTED

### 2.5. Bioenergetic Study

The glycolytic function of macrophages was measured using a Seahorse XF96 Analyzer (Agilent Technologies, USA) following the manufacturer's instructions. Extracellular acidification rates (ECAR) and oxygen consumption rates (OCR) were assessed by using Seahorse XF Glycolysis Stress Test Kit and Seahorse XF Cell Mito Stress Test Kit, respectively. Briefly, the treated macrophages were seeded at a density of 3 × 10^6^ cells per well into a Seahorse XF 96 cell culture microplate for 2 h prior to the assay. After baseline measurements, glucose, oligomycin (oxidative phosphorylation inhibitor), and 2-DG (glycolytic inhibitor) were sequentially injected into each well at indicated time points for ECAR, and oligomycin, FCCP (p-trifluoromethoxy carbonyl cyanide phenylhydrazone), and rotenone plus the antimycin A (Rote/AA) were sequentially injected for OCR. Data were assessed by Seahorse XF-96 Wave software and expressed as picomoles per minute (OCR) or miles per hour per minute (ECAR).

### 2.6. Co-Immunoprecipitation

Cells were lysed on ice by adding NP-40 Lysis Buffer for 30 min. After then, the cells were lysed at 12,000 r/min and centrifuged at 4°C for 30 min. The supernatant was collected and added with IgG and Protein A/G Plus Agarose for prewashing. The protein concentration was detected using the BCA kit (Beyotime Biotechnology, Shanghai). The lysate was divided into 2 groups, each with 1 mg protein. The IgG antibody was used as a negative control, and the Flag antibody was used as the experimental group. The cell lysate was incubated with the antibody overnight at 4°C. After 18 hours, Protein A/G agarose beads were added to incubate for 4 hours, followed by washing 5 times with NP-40 and adding to the sample. The precipitated proteins were examined using western blot analysis with the specified antibodies after the addition of 2× SDS loading buffer.

### 2.7. GST Fusion Protein Purification

The GST fusion protein pellet was transformed into E. coli Rosetta competent cells and streaked on a plate containing ampicillin antibiotics. After being cultured at 37°C overnight, a single colony was picked and inoculated in 100 mL LB liquid medium. When the OD600 absorbance reached 0.6–0.8, IPTG was added to a final concentration of 0.2 mmol/L and induced at room temperature for 4–6 h. The cells were collected by centrifugation, and the cells were lysed on ice with the lysis buffer containing protease inhibitors for 10 min, followed by ultrasonic disruption for 20 min. The supernatant was collected by centrifugation at 4°C, and DTT was added to a final concentration of 1 mmol/L according to GST Fusion Protein Spin Purification Kit (GE).

RETRACTED

### 2.8. Glutathione S Transferase (GST) Pulldown

Cells were lysed in the lysate (containing protease inhibitors) for 30 minutes on ice and centrifuged at 4°C, 12,000 r/min for 30 minutes. After then, the supernatant was collected and the protein concentration was detected using the BCA kit (Beyotime Biotechnology, Shanghai, China). The purified GST fusion protein was combined with the whole-cell lysate mix and incubated overnight at 4°C with rotation. The beads were washed 5 times with lysate, followed by adding 2× SDS buffer to the sample, and then western blotting assay was used to detect the bound proteins.

### 2.9. GEPIA Database Analysis

The co-expression level of Siglec15 and the metabolism-related gene mRNA in PDAC were analyzed by using the GEPIA database (http://gepia. cancer-pku.cn) which integrates database information such as TCGA and GTEx [20]. | log2FC | The cutoff value was set to 1, and the *p* cutoff value was 0.01. The database was also used to verify the correlation between expressions of Siglec15 and overall survival (OS) of pancreatic cancer.

### 2.10. Mice and Tumor Study

For tumor study in vivo, a single-cell suspension of Pan-02 cells (5 × 10^6^ cells) in 0.2 mL of PBS was subcutaneously injected into the right back of female WT or Siglec15 KO C57/BL6 mice aged 6 to 8 weeks. Mice were raised under specific pathogen-free (SPF) conditions at the Sir Run Run Shaw Hospital, Zhejiang University School of Medicine. Tumor growth was monitored using a vernier caliper every 5 days, and tumor volume was calculated as follows: *V* (mm^3^) = (length × width^2^) × 0.5. After four weeks, the mice were sacrificed and dissected. The overall survival of WT or Sigelc-15 ko mice were presented as days, and the survival curve was drawn. The log-rank (Mantel-Cox) test in GraphPad Prism was used for analysis. For macrophage and tumor cell co-injection model, bone marrow-derived macrophages from wild-type and Siglec-15 KO mice were extracted and cultured in vitro, followed by mixing with Pan-02 cells in single-cell suspension with a total of 1 × 10^6^ cells (mixing ratio: 1 : 1). Female wild-type mice aged 6–8 weeks were selected, and 200 *μ*L of single-cell suspension was injected into the right back subcutaneously. Subsequently, the volume of tumor was monitored every 5days. All animal experiments in this experiment have been reviewed and approved by the animal care committee of Sir Run Run Shaw Hospital, Zhejiang University.

RETRACTED

### 2.11. Statistical Analysis

Quantitative data were expressed as means with standard deviations. Means between two groups are compared using Student's *t*-test, whereas means between multiple groups are compared using one-way analysis of variance (ANOVA) with Bonferroni's post hoc test. The SNK or LSD method was used for multiple comparisons. The Kaplan-Meier method was used to generate survival curves, and the long-rank test was utilized to compare different survival rates. These analyses of overall survival were carried out. The hazard ratios (HR) and 95% confidence intervals (CIs) were calculated using a Cox regression model with two-sided Wald tests. The GraphPad Prism5 software (version 5.02, GraphPad Software, USA) was used for statistical analysis and graphing. *p* < 0.05 was considered statistically significant.

## 3. Results

### 3.1. Siglec-15 Is Expressed Differently in M1 and M2 Macrophages

IL-4 was used to polarize bone marrow-derived macrophages (BMDMs) into M2-type macrophages. Then, qPCR assay was performed for detecting Siglec family members, such as CD169, CD22, CD33, Siglec-7, Siglec-G (Siglec10), and Siglec-15, in M2-type macrophages. The results indicated that Siglec-15 was the most significantly upregulated in M2-type macrophage cells (Figure 1(a)). In addition to infiltrating many immune cells in the tumor microenvironment, the most abundant one is the tumor cells themselves. Therefore, we used qPCR assay to detect Siglec-15 expression in H6C7, SW1990, PANC-1, BXPC-3, and M2-macrophage cell lines. The results suggested that compared with pancreatic cancer cells and normal pancreatic epithelial cells, the expression of Siglec-15 was relatively much higher in M2 phenotype TAMs (Figure 1(b)), further indicating that Siglec-15 may be more important for the regulation of TAMs in human pancreatic cancer than tumor cell themselves. In addition, when using Kaplan-Meier (KM) method for univariate analysis based on TCGA data, patients with low Siglec-15 expression levels have longer overall survival (Figure 1(c)), indicating that Siglec-15 expression levels are an independent prognostic factor for the overall survival of patients with pancreatic cancer. Besides, in terms of RNA level, Siglec-15 was downregulated in M1 macrophages induced by LPS+IFN*γ* while it was upregulated in M2 macrophages induced by IL-4 or tumor supernatant (Figures 1(d)–1(f)). Simultaneously, at the protein level, the expressions of Siglec-15 as well as M2-macrophage biomarkers (CD206, Arg1) were upregulated in BMDM cells which were induced with IL-4 (Figure 1(e)). Taken together, these findings suggested that Siglec-15 might be involved in the regulation of TAMs in the TME of pancreatic cancer.

RETRACTED

### 3.2. Deletion of Siglec-15 Inhibits the Polarization of Macrophages towards M2 Macrophages

The main focus of research on TAMs in the tumor microenvironment was the polarization and phagocytosis of tumor cells, which are regulated by related genes or receptors. Previously, we found that Sigelc-15 is highly expressed in M2 macrophages. Therefore, we hypothesized whether Siglec-15 is involved in the regulation of TAM polarization. For further verification, we extracted BMDMs from WT and Siglec-15 KO mice and induced them into M1 or M2 phenotype macrophages by using LPS plus IFN-*γ* or IL-4 stimulation. In addition, for the better simulation of the effect caused by cytokines which are secreted by tumor cells on TAMs in the TME, we also collected the supernatant of pan02 cells and stimulated macrophages with tumor supernatant conditioned medium. After then, qPCR assay was performed to detect the inflammatory factors and chemokines expressed by M1 macrophages and biomarkers expressed by M2 macrophages. The results showed that knocking out Siglec-15 in macrophages does not affect biomarker genes of M1 macrophages (Figures 2(a)–2(c)) while significantly inhibiting the IL-4 (Figures 2(d)–2(f)) or Pan02 supernatant-induced M2 macrophage marker genes (Figures 2(g)–2(i)).

### 3.3. The Effect of Siglec-15 on the Glycolytic Pathway of RAW264.7 Macrophages

Metabolic changes play an important role in the activation phenotype of immune cells by regulating critical transcription and posttranscriptional events. Hence, we detected the influence of Siglec-15 on the metabolism level of RAW264.7 macrophages, hexokinase activity, and lactic acid production. The results showed that both hexokinase activity and lactate production of macrophages were significantly reduced in the macrophages which were induced with IL-4 or Pan02 supernatant (Figures 3(a)–3(d)), while knocking out Siglec-15 could significantly inhibit this phenomenon. Besides, when performing qRT-PCR (qPCR) assay to detect the changes in the mRNA transcription level of metabolic enzymes related to the glycolysis pathway, we also found that knocking down Siglec-15 significantly reduced the relative expression of metabolic enzymes which are related to the glycolysis pathway of macrophages (Figure 3(e)). These findings suggest that Sigelc-15 might upregulate the glycolysis pathway of macrophage.

RETRACTED

### 3.4. Siglec-15 Could Interact with Glut1 Directly to Regulate Macrophage Polarization

For further validation of the interaction between Siglec-15 and related downstream genes, Siglec-15 and Glut1 in RAW265.7 cells were co-expressed, followed by a immunoprecipitation experiment (Co-IP). The results revealed that Siglec-15 could interact with Glut1 (Figure 4(a)). Furthermore, we also performed a GST pulldown assay in vitro and found that Siglec-15 could directly combine with Glut1 (Figure 4(b)). That means Siglec-15 might directly interact with Glut1 to regulate the glucose metabolism. To confirm whether Siglec-15-mediated M2-type polarization of macrophages is affected by Glut1, we detected the expression of M2-type macrophage biomarkers such as Arg-1 and iNOS using qPCR and WB assay. The experimental results indicated that knocking down Glut1 could significantly overexpress the upregulated expression of Arg-1 and iNOS induced by Siglec-15 (Figure 4(c)). Taken together, these results above suggest that a direct interaction between Siglec-15 and Glut1 is involved in the regulation mechanisms of M2 phenotype macrophage polarization.

### 3.5. Siglec-15 Regulates Macrophage Inflammatory Factors Partly Dependent on STING

Glut1 is associated with the regulation of glycose metabolism and involved in response to oxidative stress. Furthermore, oxidative stress could disrupt the original balance of cytoplasmic nucleic acid metabolism and increase the nuclease tolerance of cytoplasmic DNA. These could result in DNA accumulation in the cytoplasm and activate the cGAS-STING signaling pathway to express and release associated inflammatory factors. Therefore, we continue to explore the influence of Siglec-15 on macrophage polarization regulation and the role of the cGAS-STING signaling pathway. We extracted the primary generation of peritoneal macrophages from Siglec-15-KO and wild-type mice and stimulated them with IL-4 or Pan-02 supernatant. The results show that at different time points of IL-4 stimulation, the expression of cGAS protein and phosphorylated STING in the wild-type group gradually decreased, while there was no change in the sigec-15-KO group. Besides, the stimulation of Pan-02 supernatant also had similar results (Figures 5(a) and 5(b)). In addition, cisplatin, which had been confirmed to cause the cGAS-STING signaling pathway activation in macrophages, was employed again in primary macrophages of mice with Siglec-15 overexpression and knockout. Then, we found that overexpression of Siglec-15 could reduce the activation of the cGAS-STING signaling pathway induced by cisplatin in primary macrophages, while deletion of Siglec-15 rescued the downregulated cGAS-STING signaling induced by IL-4 (Figures 5(c) and 5(d)).

RETRACTED

### 3.6. Glut1-Related Oxidative Stress Is Involved in the Regulation of Macrophage Inflammatory Factors

To confirm whether Glut1-related oxidative stress plays a role in the cGAS-STING pathway, we used BAY-876 (an inhibitor of Glut1) in further study. The results showed that in the primary peritoneal macrophages of wild-type or STING-KO mice, the phosphorylation of TBK1 decreased significantly with the stimulation of IL-4 or Pan-02, while BAY-876 could inhibit this phenomenon (Figures 6(a) and 6(b)). In addition, the transcription and released levels of M1-macrophage-related inflammatory factors such as TNF-a, IL-1*β*, and IL-6 were significantly decreased in either the WT or STING KO macrophage treated with IL-4 (Figure 6(c)), while BAY-876 could significantly inhibit this phenomenon (Figure 6(d)). These findings suggest that Siglec-15 might participate in regulating the cGAS-STING signaling pathway through Glut1-related oxidative stress.

### 3.7. Siglec-15 Knockout Inhibits the Growth of Subcutaneous Transplanted Tumors in Mice

For tumor study in vivo, we first selected 6–8-week-old WT and Siglec-15-KO C57/BL6 mice and injected Pan-02 cells subcutaneously on the back. Then, we tracked tumor growth at different time points over time and peeled off tumors and took pictures after 25 days. The results showed that the volume of subcutaneously transplanted tumors in Siglec-15 knockout mice is significantly smaller than that of WT mice (Figures 7(a) and 7(b)). Simultaneously, after constructing the animal model, we also observe the 20th day and drew a survival curve. The results revealed that absence of Siglec-15 significantly increased the survival rate of subcutaneous tumor-bearing mice (Figure 7(d)) and reduced the number of metastatic lymph nodes (Figure 7(d)). For the purpose of eliminating the interference of other cell regulations involved in Siglec-15, we mixed macrophages from WT or Siglec-15 KO mice with Pan-02 at the 1 : 1 ratio, followed by co-injecting into wild-type C57/BL6 mice on the back subcutaneously. Interestingly, we observed that the growth of tumor volume was significantly slow in the Pan − 02 + Siglec − 15 KO macrophage co-injecting model (Figures 7(e) and 7(f)). These finds further suggest that Sigelc-15 affects the tumor progression by regulating TAMs in the TME of pancreatic cancer.

## 4. Discussion

It is generally accepted that the TME plays an important role in the regulation of antitumor immunity and tumor progression including pancreatic cancer. Tumor-associated macrophages (TAMs) which are the most abundant infiltrative immune cells in the TME have a tremendous impact in the formation of an immunosuppressive tumor microenvironment [7]. Although TAMs exhibit dual functions of inducing tumors or inhibiting tumor progression according to different factors existing in the TME, they preferentially polarized into M2-like phenotype macrophages and contributed to tumor progression in various cancers, including PDAC [9–12]. In addition, it was also reported that M2-macrophage infiltration was significantly associated with chemoresistance and poor prognosis of PDAC [11, 12]. However, the mechanisms of TAM polarization are still unclear.

RETRACTED

In recent years, members of the sialic acid-binding immunoglobulin-like lectin (Siglecs) family are reported to play a critical role in regulation of immune tolerance, inflammatory response, and tumor progression of various tumors [21–23]. Among them, Sigelc-15 appears as an emerging target for tumor immunotherapy especially for patients who do not respond to PD-1/PD-L1 inhibitor treatment. Previous studies indicated that Siglec-15 is highly expressed in M2 macrophages and mainly regulates the effector T cell growth relying on the interleukin 10 (IL-10) level in the TME [24]. In addition, it was also suggested that Siglec-15 could enhance tumor immune escape in the TME without an association with the PD-1/PD-L1 pathway [13–15]. However, whether it is involved in functional regulation of macrophages in pancreatic cancer is still unclear. To address this issue, we used LPS and IFN-*γ* to induce BMDMs derived from WT or Siglec-15-KO mice into M1-type macrophages, while using IL-4 or supernatant from PANC-1 tumor cells to induce BMDMs into M2-type macrophages. Then, we performed qPCR assay to detect the expression of different biomarker genes related to macrophages. Interestingly, we found that in BMDMs derived from Siglec-15 KO mice, the expression of M2-type macrophage biomarkers such as Arg1 and CD206 was significantly decreased. These results suggest that Siglec-15 participates in the polarization process of M2-type macrophages in the TME of PDAC.

For the purpose of further investigating the biological function of Siglec-15 on macrophage and tumor progression of PDAC, we then established a series of tumor studies on mice. Then, we found that when knocking out Siglec-15 in mice, it could significantly inhibit the tumor progression of PDAC transplanted subcutaneously and improve the survival time of tumor model mice. In addition, to confirm the specific regulation of TAMs caused by Siglec-15 in PDAC, we further co-injected macrophages from WT or Siglec-15 KO mice and PANC-1 cells into WT mice aged 6–8 weeks. The experimental results showed that co-injection with macrophage from WT mice could significantly promote the tumor growth, while co-injection with Siglec-15 KO macrophages showed opposite results. Therefore, we believe that Siglec-15 could inhibit tumor progression of PDAC by regulating TAMs located in the TME.

RETRACTED

After establishing that Siglec-15 has a regulatory influence on macrophage polarization both in vitro and in vivo, we proceeded to investigate the cellular and molecular mechanisms by which Siglec-15 exerts this effect, as well as the specific role it plays in the progression of tumors. Glut1 is an important member of the glucose transporter family, which regulates glucose transport and metabolism [25]. Numerous studies have shown that a high expression of Glut1 is associated with tumor progression and poor prognosis in multiple cancer types including PDAC [26–29]. Simultaneously, it is also reported that Glut1 is involved in oxidative stress response [30]. Interestingly, in our further study we also found that deficiency of Siglec-15 could inhibit the polarization of macrophages toward M2 phenotype macrophages by downregulating metabolism-related enzymes and the extracellular acidification rate (ECAR) and oxygen consumption rate (OCR) were also significantly higher in Siglec-15 KO macrophages. That means glycolysis or metabolism-related pathway and genes might be involved in polarization-regulating mechanisms. Therefore, we further analyzed the clinical correlation between Siglec-15 and co-expressed metabolic genes using TCGA database and found that Glut1 has a strong correlation with Siglec-15. These results suggest that Glut1 might play a role in M2 phenotype macrophage polarization regulated by Siglec-15. For further validation, we also conducted the CO-IP, GST-pulldown assay, and M2 phenotype macrophage biomarkers and confirmed that Siglec-15 could increase the glycolysis by interacting with Glut1 to regulate the polarization of TAMs in PDAC.

Another interesting finding of this study was that the cGAS-STING pathway was partly involved in the regulation of macrophage inflammatory factor secretion. Cyclic GMP-AMP synthase (cGAS) was a cytosolic dsDNA sensor that triggers innate immune response via production of cGAMP, which is the adaptor protein of STING. Activation of the cGAS-STING signal pathway could promote the expression and secretion of type I interferon and inflammatory factors such as TNF-*α* and IL-6 [31]. Besides, studies have also shown that the cGAS-STING signaling pathway was critical in acute pancreatitis, autoimmune diseases, and tumors [32]. In our study, we confirmed that Siglec-15 could partly inhibit the activation of cGAS-STING and the regulation of glycolysis related to Glut1 plays a role in this process.

RETRACTED

However, the present study had several limitations. First, the expression of Siglec-15 in PDAC patients was not confirmed and further confirmation using more tumor samples is needed to confirm the expression and diagnostic value of Siglec-15 in PDAC patients. Second, although we found that a high Siglec-15 expression was associated with poor prognosis in PDAC patients based on TCGA datasets, its prognostic value in other cohort was not confirmed. Third, the potential mechanisms involved in the function of Siglec-15 regulating the inflammatory response needed to be further studied.

Taken together, our data suggested that Siglec-15 was critical for the polarization of TAMs in PDAC. It could interact with Glut1 and inhibit the cGAS-STING pathway in regulation of TAM polarization and release of the macrophage inflammatory factor to promote the tumor progression of PDAC. Hence, our findings were expected to provide a novel immunotherapy strategy for the patients with PDAC.

## Figures and Tables

**Figure 1:** Siglec-15 was expressed differently in M1 and M2 macrophages. (a) 20 ng/mL IL-4 was used to induce MФ into M2 type. The expression of the Siglec family in M2-type MФ was detected by qPCR. (b) Extract the total RNA of different tumor cells and TAMs and use qPCR assay to detect the expression level of Siglec-15. (c) Correlation analysis between the expression level of Siglec-15 and the overall survival (OS) of pancreatic tumors. (d) Siglec-15 transcription level of BMDMs stimulated by 100 ng/mL LPS and 20 ng/mL IFN-*γ*, or 20 ng/mL IL-4. (e) Siglec-15 protein level of BMDMs stimulated by 100 ng/mL LPS and 20 ng/mL IFN-*γ*, or 20 ng/mL IL-4. The experiments were repeated three times, and each experiment was triplicated.

**Figure 2:** Deletion of Siglec-15 inhibits the polarization of macrophages towards M2. (a–c) Bone marrow cells from wild-type and Siglec-15 knockout mice were extracted in vitro and induced into bone marrow-derived macrophages (BMDMs). 100 ng/mL LPS and 20 ng/mL IFN-*γ* to stimulate for 12 hours; induce them into M1-type macrophages and detect the inflammatory factors expressed by M1-type macrophages by qPCR. (d–f) 20 ng/mL IL-4 to stimulate BMDMs cells for 24 h or 48 h to induce into M2-type macrophages. qPCR detects the marker genes expressed by M2-type macrophages. (g–i) Tumor supernatant conditioned medium to stimulate BMDM cells for 24 h or 48 h to induce into M2-type macrophages, and qPCR to detect the marker genes expressed by M2-type macrophages. The experiments were repeated three times, and each experiment was triplicated.

RETRACTED

**Figure 3:** The effect of Siglec-15 on the glycolytic pathway of RAW264.7 macrophages. (a) Bone marrow cells from wild-type and Siglec-15 knockout mice were extracted in vitro and induced into bone marrow-derived macrophages (BMDMs). The effect of IL-4 stimulation on ECAR of BMDMs cells. (B) The effect of IL-4 stimulation on the ECAR of BMDMs cells. (c) The effect of IL-4 stimulation on the lactic acid production of BMDMs cells. (d) The effect of IL-4 stimulation on HK enzyme activity. (e) The effect of Siglec-15 knockout of RAW264.7 and BMDMs on the transcription level of glycolysis-related genes.

**Figure 4:** Siglec-15 interacts with Glut1 to regulate macrophage polarization. (a) Immunoblotting of cell lysate co-transformed with Siglec-15-FLAG+Glut1-HA with FLAG antibody immunoprecipitation. (b) GST protein pulldown results of GST/GST-Glut1 protein and Glut1 protein. (c) qPCR assay indicated that knocking down Glut1 can overexpress Siglec-15-induced upregulation of Arg1 expression which was a biomarker of M2 phenotype macrophage. (d) Western blotting assay indicated that knocking down Glut1 can overexpress Siglec-15-induced upregulation of Arg1 expression which was a biomarker of M2 phenotype macrophage. (e) qPCR assay indicates that knocking down Glut1 can overexpress Siglec-15-induced upregulation of iNOS which is another biomarker of M2 phenotype macrophage. (f) Western blotting assay indicate that knocking down Glut1 can overexpress Siglec-15-induced upregulation of iNOS which is another biomarker of M2 phenotype macrophage. The experiments were repeated three times, and each experiment was triplicated.

**Figure 5:** Siglec-15 regulates macrophage inflammatory factors partly dependent on STING. (a) BMDMs of bone marrow-derived macrophages from WT and Siglec-15 KO mice were extracted, and 50 ng/mL IL-4 stimulated the cells. The proteins were collected according to different experimental time points, and the cGAS-STING signaling pathway was detected by western blot. (b) BMDMs of bone marrow-derived macrophages from WT and Siglec-15 KO mice were extracted, and conditioned medium containing Pan-02 supernatant stimulated the cells. The proteins were collected according to different experimental time points, and the cGAS-STING signaling pathway was detected by western blot. (c) After extracting Sigle-15KO mouse peritoneal primary macrophages, stimulated with cisplatin for 24 hours, the protein expression of the cGAS-STING signaling pathway conditioned medium containing Pan-02 supernatant was as shown in the figure. (d) After extracting Sigle-15KO or Sigle-15 OE mouse peritoneal primary macrophages, after IL-4 stimulation, the expression of cGAS-STING signaling pathway molecule protein-conditioned medium containing Pan-02 supernatant was as shown. The experiments were repeated three times, and each experiment was triplicated.

RETRACTED

**Figure 6:** Glut1-related glycolysis is involved in regulating macrophage inflammatory factors. (A) The peritoneal macrophages of wild-type and STING-KO mice were separately extracted and pre-incubated with Bay-876 for 30 minutes. After stimulation with IL-4, the expression of the cGAS-STING signaling pathway molecules changed. (b) The peritoneal macrophages of wild-type and STING-KO mice were extracted separately and pre-incubated with Bay-876 for 30 minutes. After stimulation with Pan-02 supernatant, the expression of cGAS-STING signaling pathway molecules changed. (c, d) After the above stimulation, the transcription level and release changes of inflammatory factors related to M1-macrophage were detected. The experiments were repeated three times, and each experiment was triplicated.

**Figure 7:** Siglec-15 knockout inhibits the growth of subcutaneous transplanted tumors in mice. (a, b) Six to 8 weeks of wild-type and Siglec-15 KO mice, 200 *μ*L of tumor cells was injected subcutaneously, the tumor volume was calculated and statistics (*n* = 10), and the tumor was peeled off and photographed. (c) In the survival curve experiment, the survival of mice was observed and recorded every day from the 20th day (*n* = 14). (d) Take mouse lymph nodes and count the tumor nodules in the lymph nodes. (e, f) Six- to 8-week-old wild-type mice were selected for macrophage and tumor cell co-injection model (200 *μ*L, 1 : 1). The tumor was measured once in 5 days for recording and stripped and photographed. ∗*p* < 0.05; ∗∗*p* < 0.01; ∗∗∗*p* < 0.001. The experiments were repeated three times, and each experiment was triplicated.

**Table 1:** The primer sequences included in this study.

Name	Primer sequences (5′–3′)
Siglec-15: forward	GTTCTCGGGCACCTTGG
Siglec-15: reverse	AGCTCCGAAATGGTTGTCC
NOS2: forward	TTCAGTATCACAACCTCAGCAAG
NOS2: reverse	TGGACCTGCAAGTTAAAATCCC
IL-6: forward	TCCATCCAGTTGCCTTCTTGG
IL-6: reverse	CCACGATTTCCCAGAGAACATG
Arg-1: forward	CTTCAGAGAAGTGGCCCAAC
Arg-1: reverse	GGTGGTGGGTATCACAGGAC
TNF-*α*: forward	AG CAAACCACCAAGTGGAGGA
TNF-*α*: reverse	GCTGGCACCACTAGTTGGTTGT
GAPDH: forward	ACCCAGAAGACTGTGGATGG
GAPDH: reverse	CACATTGGGGGTAG GAACAC
U6: forward	GCGCGTCGTGAAGCGTTC
U6: reverse	GTGCAGGGTCCGAGGT

## Data Availability

The authors declare that all the other data supporting the findings of this study are available within the article and from the corresponding author upon reasonable request.
